RETRACTED

# Analysis of the Reform Effectiveness of Vocational Skill Identification Based on the New Social Training Model in the New Era under Deep Learning Assessment

**DOI:** 10.1155/2022/1676355

**Published:** 2022-03-20

**Authors:** Yeming Wang, Yong Ran

**Affiliations:** ^1^Graduate School, Anyang University, Anyang-si 14028, Gyeonggi-do, Republic of Korea; ^2^School of Intelligent Manufacturing, Chongqing Three Gorges Vocational College, Chongqing 404155, China

## Abstract

In order to be able to make full use of domain knowledge to improve the performance of skill word extraction, this paper proposes a skill word extraction method based on a combination of deep learning and corpus features. Skill word extraction is transformed into a sequence annotation problem, and based on the basic model of sequence annotation, Bi-LSTM-CRF, corpus features are added to the input layer, and the output of the input layer is connected with the Bi-LSTM output as the input of the CRF layer. The experimental results show timely updating of the question bank, paying attention to the quality of vocational skill identification, and strictly managing the issuance of vocational qualification false certificates.

## 1. Introduction

Vocational skill appraisal is an assessment activity based on the level of vocational skills belonging to the standard-referenced examination [1]. It is an objective measurement and evaluation of the technical theoretical knowledge and practical operation ability that workers should master to engage in a certain occupation by the examination and assessment institution [2].

Although China has widely popularized vocational skill appraisal, there are some problems in its implementation, and the recognition of vocational qualification certificates is low [3]. Although the county vocational skill identification work has made significant development in recent years, the community's awareness of vocational qualifications is still very low. Most of the technical personnel generally have the ability to practice the phenomenon of low cultural quality; a considerable part of the practitioners do not know what is access to employment and vocational qualification certificate system [4, 5].

A good business environment is created on the grounds that interfere with human resources and social security departments to implement the occupational qualification certificate system of labor inspection of employers resulting in passive labor inspection work, to a certain extent affecting the development of vocational skill identification work [6].

With the continuous development of science and technology, culture and economic progress of vocational skill identification requirements are also increasingly high, which inevitably makes the original library of questions not meeting the needs of vocational skill identification in a certain extent affecting the development and improvement of vocational skill identification work; especially, the emergence of some new types of jobs makes the county library of professional skill knowledge assessment not comprehensive, seriously affecting the results of the assessment and quality, so the library of questions should be improved and expanding the amount of knowledge covered by it is imperative [7].

RETRACTED

The vocational qualification certificate system is an inherent requirement for workers to realize their self-worth, which is an urgent need for enterprises to enhance their competitiveness and a fundamental task to promote the transformation of economic growth. Therefore, we should promote the employment access system and vocational qualification certificate system in a multimedia way so that more workers and employers are familiar with the relevant system through active publicity to guide the majority of workers and employers to consciously comply with the employment access system to participate in vocational skill identification [8, 9].

The strength of labor supervision is increased. Adjustment and enrichment of labor inspectors are made to increase supervision and inspection efforts, to hold a professional qualification certificate as a regular work of labor inspection [10]. The units and practitioners who ignore the legal provisions of the inspection will be firmly punished to improve the authority of vocational qualification certificates.

With the development of society, the requirements for vocational skill identification are getting higher and higher, so the disadvantages of the question bank are increasingly prominent [11], to effectively develop new questions to break through the original limitations of the organization of experts to regularly discuss and exchange, discuss the editing, and review and revise vocational skill identification test questions to carry out a new reform to understand the growth of each type of work and the development trend to meet the rapid development of society and its subtle application to the development of vocational skill identification question bank and innovation work [12].

In short, we need to address the problems that arise in the process of vocational skill identification in our county to increase the publicity and supervision of vocational skill identification to strengthen the construction of weak links and timely update the question bank to pay attention to the quality of vocational skill identification and strict management of the issuance of vocational qualifications to promote the steady development of society and improve people's quality of life [13].

RETRACTED

## 2. Deep Learning-Based Skill Word Extraction Model

The proposed skill word extraction model is shown in Figure 1. The model consists of four levels of modules, i.e., input layer, Bi-LSTM layer, feature stitching layer, and CRF layer. In the input layer, each input utterance is converted into a series of character feature vectors, then stitched with the position features (Seg) of each character in the input utterance, the lexical features (Pos), and the context features (Con) of the skill words after the input utterance is divided into words, and input them into the Bi-LSTM layer to encode the context information sequentially into a fixed-length hidden vectors, and then, the output of the input layer is connected with the output of the Bi-LSTM layer in the feature splicing layer as the input of the CRF layer. Finally, the best label sequence is predicted by the CRF layer as the output of the whole network.

### 2.1. Input Layer

The input layer is divided into 2 steps:

1. Convert the input utterance into a sequence of character-level dense vectors. The dictionary containing all the characters in the corpus is generated, and then, an embedding matrix *M* ∈ *R*^*D*×*V*^ is used to map each character into a dense vector, where *D* is the dimension of the embedding vector and *V* is the total number of all characters in the dictionary. The input sentence is represented as *S* = [*w*_1_, *w*_2_, ⋯, *w*_*n*_], where *n* is the length of the sentence and *w*_*i*_ ∈ *R*^*V*^ is the one-hot representation of the *i*th character in the dictionary. The character embedding vector of the sentence is denoted as [*c*_1_, *c*_2_, ⋯, *c*_*n*_], where *C*_*i*_ ∈ *R*^*D*^
2. Add various corpus features of characters in online job information and splice with the character embedding vector. The corpus features are mainly composed of three kinds of features: position features (Seg), lexical features (Pos), and context features (Con)

The position feature (Seg) is the relative position of each character to the word in the input sentence after the jieba splitting. For example, if “operation system” is the word obtained after splitting, the location feature of “operation” is marked as “0,” the location feature of “operation” is marked as “0,” the location feature of “operation” is marked as “1,” the location feature of “system” is marked as “2,” and the location feature of “system” is marked as “1.” The position feature of “system” is marked as “2,” and the position feature of “unified” is marked as “3.” The lexical feature (Pos) is the lexical character of each character that is marked as the corresponding lexical character of the word in the input statement after the jieba division. For example, if the lexical property of “have” is “verb,” then the lexical properties of “have” and “ready” are both recorded as “verb.” As we can see from the characteristics of the terminology, some words only circulate in this field.

RETRACTED

Contextual features (Con) are features constructed based on the contextual characteristics of skill words. First, we analyzed the recruitment corpus and randomly selected more than 1,000 online recruitment texts and found that the texts containing skill words are usually in verb-object structures, and most of the skill words are “nouns/noun phrases,” such as “familiar with relational database.” The position of the skill word in the sentence is mainly after the verb, adjective/phrase or “and,” “or” and “,” etc., for example, “understand natural language processing,” “commonly used machine learning algorithms,” “master text mining, entity extraction, lexical annotation, and other techniques.” Table 1 shows the positions of skill words in the online recruitment corpus. By analyzing the context in which the skill words appear, we can find that more idioms are used in the context, such as “mastering XX ability” and “having XX experience.”

Therefore, when labeling the context features, the input utterances are firstly subdivided by jieba to extract the lexical properties of each word and then labeled according to the following rules.

Finally, the output of the input layer consists of four sets of feature vectors: character feature vector, position feature vector (Seg), lexical feature vector (Pos), and context feature vector (Con) for each node in each input statement sequence, i.e., **X**_*i*_ = [ci, segi, coni]. For example, if the input statement is “with database and data structure foundation,” the lexical feature vectors are “0, 0, 1, 1, 1, 1, 2, 1, 1, 1, 1, 1, 1, 1,” where “0 “represents verbs, “1” represents nouns, and “2” represents conjunctions. The location feature vector is expressed as “0, 1, 0, 1, 2, 0, 0, 1, 2, 3, 0, 1”, where “0” represents the first character of the word, “1” represents the second character of the word,…. Contextual features are expressed as “1, 1, 0, 0, 0, 0, 3, 0, 0, 0, 0, 0, 4, 4.”

### 2.2. Bi-LSTM Layer

LSTM is a special type of recurrent neural networks (RNN) that can capture long-range sequence information and is powerful in modeling sequence data. The difference from the standard RNN is that LSTM adds cell states and input gates, forgetting gates, and output gates to the neurons in the hidden layer. The cell states are updated by using both the input gate and the forgetting gate results. The specific implementation is

(1) $$\begin{array}{c} i_{t}=\sigma \left(W_{xi}V_{t}+W_{hi}h_{t-1}+W_{ci}c_{t-1}+b_{i}\right), \end{array}$$

(2) $$\begin{array}{c} f_{t}=\sigma \left(W_{xf}X_{t}+W_{hf}h_{t-1}+W_{cf}c_{t-1}+b_{f}\right), \end{array}$$

(3) $$\begin{array}{c} c_{t}=f_{t}⊗c_{t-1}+i_{t}⊗\tanh\left(W_{xc}X_{t}+W_{hc}h_{t-1}+b_{c}\right), \end{array}$$

(4) $$\begin{array}{c} o_{t}=\sigma \left(W_{xo}X_{t}+W_{ho}h_{t-1}+W_{cc}c_{t}+b_{o}\right), \end{array}$$

(5) $$\begin{array}{c} h_{t}=o_{t}⊗\tanh\left(c_{t}\right), \end{array}$$

where *σ* is the logistic sigmoid activation function and ⊗ is the product of elements. At moment *t*, *i*, *f*, *o*, and *c* represent the input gate, the forgetting gate, the output gate, and the cell state, respectively. The input gate, output gate, and forgetting gate are implemented by the sigmoid activation function, and the cell state is controlled by the three gates. The subscript of the weight matrix *W* represents the connection between each gate, and *b* is the bias. For example, **W**_*xi*_ is the weight matrix between the input node **X**_*t*_ and the input gate, **W**_*hi*_ is the weight matrix between the hidden layer state **h**_*t*−1_ and the input gate at moment *t* − 1, and **W**_*ci*_ is the weight matrix between the cell state **c**_*t*−1_ and the input gate at moment *t* − 1.

RETRACTED

### 2.3. Feature Splicing Layer

The feature stitching layer stitches the output of Bi-LSTM with the character embedding feature vector, position features (Seg), lexical features (Pos), and skill word context features (Con) in the previous input layer, in order to better improve the recognition accuracy of the model. After the splicing, the feature of the *i*th character is represented as **A**_*i*_ = [**h**_*i*_, **X**_*i*_], where **X**_*i*_ is the output of the *i*th character in the input layer and **h**_*i*_ is the output of the *i*th character in the Bi-LSTM layer. In addition, in order to avoid simple linear combination and enhance the nonlinear factor of the neural network model, it is proposed to map the vector **A**_*i*_, which is the output of the Bi-LSTM layer and the input layer after stitching, into an *L*-dimensional vector before the output of the feature stitching layer, where *L* is the number of tags in the skill word tag set. That is, **O**_*i*_ = tanh(*w*∗**A**_*i*_ + *b*), *O*_*i*_ ∈ **R**^*L*^, where tanh is the activation function, *w* is the weight of the mapping, *b* is the bias, and *φ* = {*w*, *b*} is denoted as the parameter set in the feature splicing layer. Finally, the output of the feature splicing layer is **O** = [**O**_1_, **O**_2_, ⋯, **O**_*n*_].

RETRACTED

### 2.4. CRF Layer

Denote the sequence of tags of sentence *S* by *y* = [*y*_1_, *y*_2_, ⋯, *y*_*n*_], where *y*_*i*_ ∈ *R*^*L*^ is the one-hot representation of the *i*th character tag. The input of the CRF layer is the output of the feature splicing layer, and the output of the CRF layer is the sequence of tags *y*. The conditional probability of the sequence of tags *y* for input *O* is calculated as follows [14]:

(6) $$\begin{array}{c} p\left(\left.y\right|O,\theta \right)=\frac{\prod_{i=1}^{n}\Psi \left(O_{i},y_{i},y_{i-1}\right)}{\sum_{y^{\prime }\in Y\left(S\right)}\prod_{i=1}^{n}\Psi \left(O_{i},y_{i}^{\prime },y_{i-1}^{\prime }\right)}, \end{array}$$

where *Y*(*S*) is the set of all possible sequences of labels for sentence *s* and Ψ(**O**_*i*_, **y**_*i*_, **y**_*i*−1_) is the potential function:

(7) $$\begin{array}{c} \Psi \left(O_{i},y_{i},y_{i-1}\right)=e^{\left(y_{i}^{T}E^{T}o_{i}+y_{i-1}^{T}F_{y_{i}}\right)}, \end{array}$$

where **E** ∈ **R**^*L*×*L*^, **F** ∈ **R**^*L*×*L*^ is the parameter of the CRF layer and *θ* is the parameter set, i.e., *θ* = {*E*, *F*}. The loss function of the CRF layer

(8) $$\begin{array}{c} f_{\text{Loss}}=-\underset{s\in \text{corpus }}{\sum }\log\left(p\left(\left.y_{S}\right|O_{S},\theta \right)\right), \end{array}$$

where corpus is all statements in the training dataset.

## 3. Experimental Results and Analysis

### 3.1. Experiment 1

This set of experiments was conducted to verify the effects of the various types of corpus features incorporated in the proposed skill word extraction model on the effectiveness of skill word extraction. The specific experimental setup is as follows: the character-level Bi-LSTM-CRF model is chosen as the baseline comparison experiment, at which time only the characters are embedded in the feature input network and no corpus features of the characters are input.

Then, different types of corpus features are added to the input layer of the Bi-LSTM-CRF model, e.g., Model_1 represents the addition of character location features (Seg) to the input layer of the Bi-LSTM-CRF but not the output of the Bi-LSTM-CRF model. The output of the output layer is not spliced with the output of the Bi-LSTM layer, and Model_4 represents the addition of the contextual features of skill words (Con) to Model_1, i.e., the addition of all corpus features to the input layer of Bi-LSTM-CRF. Model_8 represents the addition of all corpus features in the input layer of Bi-LSTM-CRF and the splicing of the output of the output layer with the output of the Bi-LSTM layer, i.e., the final skill word extraction model.

As can be seen from Table 2, when the location features (Seg), lexical features (Pos), and contextual features of skill words (Con) are added to the input layer of the Bi-LSTM-CRF model, the F1 values increase by 0.44%, 0.35%, and 7.66%, respectively, compared with those of the Bi-LSTM-CRF model. The F1 values are increased by 0.44%, 0.35%, and 7.66%, respectively, compared with the Bi-LSTM-CRF model. This is because the syntactic structure of the recruitment corpus is relatively single and the contextual features of skill words are relatively fixed, so the full exploitation of the contextual features of skill words can better reflect the position of skill words in the corpus and can effectively extract “… with database development ability …” “… common programming languages such as Java, C, python …” such skill words with obvious syntactic structure, thus making the trained model more generalizable. The addition of positional features (Seg) and lexical features (Pos) of characters, on the other hand, improves the F1 value, but the improvement is not very large. One of the possible reasons is that the word position feature (Seg) is obtained by performing jieba word separation on the sentence and then extracting the relative position of each character and the word it is in. The inaccuracy of the Chinese word separation results affects the extraction of character position features, thus causing a certain degree of interference in the extraction of skill words. For the lexical features (Pos), it may be due to the inability of the jieba subword to label the lexical properties of English characters and the low regularity of the composition of skill words in terms of lexical features.

RETRACTED

It can also be seen from Table 2 that if both positional features (Seg) and lexical features (Pos) of characters are added to the input layer of the Bi-LSTM-CRF model, the F1 value of the model is improved by 0 compared to Bi-LSTM-CRF. The F1 value of the model is improved by 0.5% compared to Bi-LSTM-CRF if both the position feature of the character (Seg) and the context feature of the skill word (Con) are added to the input layer of the Bi-LSTM-CRF model and by 7.83% compared to Bi-LSTM-CRF. If both lexical features (Pos) and contextual features of skill words (Con) are added to the input layer of the Bi-LSTM-CRF model, the F1 value of the model increases by 7.83% compared to that of the Bi-LSTM-CRF. If the position feature (Seg), the lexical feature (Pos), and the context feature (Con) of the technical word are added into the input layer of the Bi-LSTM-CRF model, the F1 value of the model can be further improved from 0.789 2 to 0.870 6, which is 8.14%. The improvement is 8.14%. Therefore, the more corpus features are added to the model, the more beneficial the model is for skill word extraction.

RETRACTED

In addition, while adding all corpus features to the input layer of Bi-LSTM-CRF, the output of the input layer and the output of the Bi-LSTM layer are spliced together, which is the final proposed skill word extraction model. Compared with the case of adding only corpus features, the F1 value of the model is further improved by 8.23%. Finally, it can be concluded that the model can effectively perform skill word extraction, and the extraction performance is greatly improved, and the addition of various corpus features is also beneficial to the improvement of skill word extraction performance [15].

### 3.2. Experiment 2

In order to verify whether the various corpus features added to the model can improve the extraction performance under different sizes of training sets and to evaluate whether the rich corpus features added can alleviate the reliance of the model on a large amount of labeled data, based on Experiment 1, further samples of 25%, 50%, and 75% were extracted from the training set, while keeping the test set unchanged, and the experimental results are shown in Table 3.

The sample was extracted as follows: after dividing the data in two rounds of cross-validation, the training data were divided into *N* equal parts, and a few of them were selected as the final training set each time, and the experiment was repeated several times. For the 50% training set extraction scheme, the training set was divided into 2 copies, and 1 copy was selected as the final training set each time, and the experiment was repeated 2 times; for the 75% training set extraction scheme, the training set was divided into 4 copies, and 3 copies were selected as the final training set each time, and the experiment was repeated 4 times. In this group of experiments, the Bi-LSTM-CRF model is also selected as the baseline comparison experiment under different training set proportions [16].

As shown in Table 3, the extraction performance of this model is still improved compared with that of the Bi-LSTM-CRF model under different training set sizes, and the F1 values increase from 0.7267, 0.7646, and 0.780 7 to 0.8336, 0.8337, and 0.8647 for 25%, 50%, and 75% training sets, respectively. In addition, the inclusion of various types of corpus features at different proportions of the training set is still beneficial to the model extraction performance, and the same conclusion can be drawn as in Experiment 1 using the full training set, i.e., the more corpus features are included in the model, the more beneficial the model is to skill word extraction. For example, adding only lexical features (Pos) at 25%, 50%, and 75% of the training set increases the F1 values by 0.74%, 0.18%, and 0.48%, respectively, compared to the Bi-LSTM-CRF model. The F1 values of the Bi-LSTM-CRF model increased by 1.32%, 0.44%, and 0.46%, respectively, when both the position feature (Seg) and the lexical feature (Pos) were added to the input layer of the Bi-LSTM-CRF model and 0.46%, respectively. The F1 values of the Bi-LSTM-CRF model are further improved by adding the position feature (Seg), the lexical feature (Pos), and the context feature (Con) to the input layer of the Bi-LSTM-CRF model, from 0.7267, 0.7646, and 0.7807 to 0.8267, 0.8267, and 0.7807, respectively. The F1 values of the model can be further improved from 0.7267, 0.7646, and 0.7807 to 0.8267, 0.8491, and 0.8623, with the improvement rates reaching 10.0%, 8.45%, and 8.16%, respectively.

RETRACTED

Table 3 also shows that adding rich corpus features to the input layer of the Bi-LSTM-CRF model does alleviate the lack of available labeled data. For example, the F1 value for the input layer of the Bi-LSTM-CRF model with only character embedding features is 78.07% for a training set ratio of 75%, while the F1 value for the input layer of the Bi-LSTM-CRF model with a training set ratio of 50% is 78.07% for the input layer of the Bi-LSTM-CRF model with only character embedding features. The F1 value for the input layer of the Bi-LSTM-CRF model with the addition of positional features (Seg) and lexical features (Pos) is 76.90%; the F1 value for the input layer of the Bi-LSTM-CRF model with only character embedding features is 78.92% when the proportion of the training set is 100%, while the proportion of the training set is only 25%, and the F1 value for the input layer of the Bi-LSTM-CRF model with only character embedding features is 78.92% when the proportion of the training set is only 25%. The F1 value of the Bi-LSTM-CRF model is 81.72% when the input layer of the Bi-LSTM-CRF model uses only the contextual features of the skill words (Con), while the F1 value of the Bi-LSTM-CRF model is 81.72% when the proportion of the training set is only 25%. Therefore, it can be concluded that adding rich corpus features to this model can alleviate the reliance of the model on a large amount of labeled data [17].

### 3.3. Experiment 3

To illustrate the effectiveness of the proposed skill word extraction model, the currently dominant sequence annotation models BERT-Bi-LSTM-CRF and IDCNN-CRF models were selected for comparison. Although the comparison method chosen for this model achieves good results for experiments on English datasets, this type of framework is generic, is less affected by language differences, and uses the same data processing approach when conducting experiments [17, 18].

RETRACTED

The same experimental scheme of cross-validation is used for the partitioning of the dataset. The Bi-LSTM-CRF model is also selected as the baseline comparison model, and the experimental results are shown in Table 4. The hyperparameters of the BERT-Bi-LSTM-CRF model in Method 1 are set as follows: the initial learning rate is 0.001, the epoch number is 50, the hidden layer dimension is 100, and the batch training sample size is 32. The hyperparameters of the IDCNN-CRF model in Method 2 are set as follows: character embedding dimension is 100, initial learning rate is 0.001, epoch number is 100, convolutional kernel size is 1∗3, and batch training sample size is 20.

As can be seen from Table 4, the F1 values of the present skill word extraction model are much better than those of the BERT-Bi-LSTM-CRF model of Method 1 and the IDCNN-CRF model of Method 2. In addition, considering that the training of the BERT model uses a very large training corpus of public resources, the training of the present skill word extraction model uses only a small portion of the manually annotated corpus. Therefore, it can be concluded that the present skill word extraction model can extract skill words effectively and the incorporated corpus features are more beneficial to the extraction performance of the model [19].

## 4. Discussion

The main task of the development of the vocational qualification system is, firstly, to create productive career paths for the growth of workers and, secondly, to secure the skilled workers needed for the development of the national economy. In order to adapt to the rapidly changing technical and organizational needs of industry and to ensure the continuous updating of professional qualifications, the development of this system must always be oriented to the needs of employment and centered on the needs of industry and labor. This is the basic way to come from the enterprise and go to the enterprise; to implement the norms, solve problems, and accomplish tasks, this is the basic standard.

The technical principle of occupational classification in China is based on the homogeneity of the nature of work. For specific occupations, the homogeneity of work nature can be deduced from the homogeneity of work ability requirements of workers in industrial sites. The structure of occupational classification is an important basis for understanding the structure of occupational competence.

When comparing different occupations in the same industry together, it is found that some parts of them overlap and the common requirements within the industry are found, which we call industry generic skills, such as the generic management skills that have been developed. When the requirements of different industries are compared together, some more general requirements are found. They have universal applicability and also have a wide range of transferability. This is often overlooked. We call this level of occupational competence the core skills that form the basis of occupational competence and are essential for occupational expansiveness. The core skill criteria we are developing include personal skills such as communication skills, self-improvement and use of foreign languages, methodological skills such as innovation, problem-solving and use of numbers, and social skills such as cooperation with others and information processing [19–22].

RETRACTED

## 5. Conclusions

With the development of society, the requirements for vocational skill assessment are becoming more and more demanding. The disadvantages of the question bank are therefore becoming more and more obvious, so it is imperative to improve the question bank and expand the amount of knowledge it covers. In this paper, we propose a skill word extraction method based on the combination of deep learning and corpus features. The experimental results show that timely updating of the question bank, paying attention to the quality of vocational skill identification, and strict management of the issuance of vocational qualification certificates will promote the steady development of society and improve people's quality of life.

## Figures and Tables

**Figure 1:** Deep learning-based skill word extraction model.

**Table 1:** Location of skill words occurring in the online recruitment corpus.

Number of corpora	Number of skill words	After verb	After adjective/adjective phrase	“And,” “or, ·,” and other parallel forms	Other locations
1005	8125	2374	1925	2851	567

**Table 2:** Performance of skill word extraction after the addition of various corpus features.

Model number	Model features	Precision	Recall	F1	Promote
Model 0	Bi-LSTM-CRF	0.789	0.7894	0.7861	—
Model 1	Model 0+Seg	0.7898	0.7956	07935	+0.42%
Model 2	Model 0+Pos	0.7914	0.7951	0.7926	+0.32%
Model 3	Model 0+Con	0.7900	08655	0.7962	+0.72%
Model 4	Model 0+Con	0.8674	0.8674	0.8654	+0.75%
Model 5	Model 0+Seg+Con	0.8661	0.8665	0.8547	+0.83%
Model 6	Model 0+Seg+Pos	0.8662	0.7985	0.8479	+0.5%
Model 7	Model 0+Seg+Pos+Con	0.8714	0.7541	0.8701	+0.81%
Model 8	This skill word extraction model	0.8714	0.7524	0.8714	+0.83%

**Table 3:** Skill word extraction performance after adding various types of corpus features with different training set ratios.

Model	Training set proportion		
	25%	50%	75%
	Precision, recall, F1, lifting	Precision, recall, F1, lifting	Precision, recall, F1, lifting
Model 0	0.714, 0.7402, 0.7267	0.7549, 0.775, 0.7646	0.7769, 0.7848, 0.7807
Model 1	0.7234, 0.7512, 0.7367, +1.00%	0.7641, 0.7783, 0.7685, +0.42%	0.7841, 0.7882, 0.7859, +0.52%
Model 2	0.7195, 0.75, 0.7341, +0.74%	0.7573, 0.7761, 0.7664, +0.18%	0.7831, 0.7883, 0.7855, +0.48%
Model 3	0.8124, 0.8244, 0.8172, +0.95%	0.8131, 0.8457, 0.8433, +7.87%	0.8511, 0.8567, 0.8532, +7.76%
Model 4	0.8155, 0.8293, 0.8221, +9.54%	0.8451, 0.8539, 0.8489, +8.43%	0.8616, 0.8552, 0.8583, +7.6%
Model 5	0.8157, 0.8223, 0.8191, +1.23%	0.8443, 0.8437, 0.8467, +8.15%	0.8563, 0.8564, 0.8567, +7.6%
Model 6	0.7254, 0.7563, 0.7398, +1.32%	0.7631, 0.7775, 0.7698, +0.44%	0.7818, 0.7891, 0.7852, +0.46%
Model 7	0.8195, 0.8341, 0.8236, +10%	0.8457, 0.8562, 0.8432, +8.45%	0.8634, 0.8617, 0.8623, +8.12%
Model 8	0.8291, 0.8382, 0.8335, +10.7%	0.8491, 0.8534, 0.8517, +8.17%	0.8624, 0.8647, 0.8646, +8.38%

RETRACTED

**Table 4:** Comparison of extraction performance of different network models.

Model	Pre	Recall	F1	Promote
Bi-LSTM-CRF	0.798	0.7888	0.7891	—
Bi-LSTM-CRF	0.8155	0.8186	0.816	+2.76%
IDCNN-CRF	0.8047	0.7966	0.8008	+1.16%
Skill word extraction model	0.8705	0.8726	0.8714	+8.22%

## Data Availability

The dataset used in this paper is available from the corresponding author upon request.
